This article has been retracted.

# Ultrasound Image Features under Decomposition Algorithm to Analyze the Nursing Intervention on Patients with Colon Polyps Undergoing Endoscopic Resection

**DOI:** 10.1155/2021/9581568

**Published:** 2021-12-15

**Authors:** Na Ma, Xiujie Wang, Xinxin Zhao, Xuehan Zhao, Lin Liu

**Affiliations:** ^1^Department of Gastroenterology, Affiliated Hongqi Hospital of Mudanjiang Medical University, Mudanjiang City, 157011 Heilongjiang Province, China; ^2^Academic Affairs Section, Affiliated Hongqi Hospital of Mudanjiang Medical University, Mudanjiang City, 157011 Heilongjiang Province, China

## Abstract

Based on the ultrasonic imaging and endoscopic resection of the intelligent segmentation algorithm, this study is aimed at exploring whether nursing intervention can promote the good recovery of patients with colon polyps, hoping to find a new method for clinical treatment of the colon polyps. Patients with colon polyps were divided into an experimental group (fine nursing) and a control group (general nursing). The colonoscopy polyp ultrasound image was preprocessing to select the seed points and background points. The random walk decomposition algorithm was applied to calculate the probability of each marked point, and then, the marked image was outputted. The accuracy of the intelligent segmentation algorithm was 81%. The incidence of complications in the experimental group was 4.83%, which was lower than 16.66% in the control group, and the difference was statistically obvious (*P* < 0.05). Perioperative refined nursing intervention for colon polyp patients undergoing endoscopic electrosurgical resection can decrease postoperative adverse reactions; reduce postoperative mucosal perforation, blood in the stool, abdominal pain, and small bleeding; lower the incidence of postoperative complications; and allow patients to recover quickly, enhancing the life comfort of patient.

## 1. Introduction

A colon polyp is a common disease in clinical gastrointestinal diseases [1]. The incidence is high, and the chance of cancer is high [2]. If it is not detected in time and effective treatment measures are taken, it will seriously threaten the life safety of patients [3]. At present, the clinical treatment mainly adopts endoscopic high-frequency electrocoagulation and resection, and the clinical effect is significant [4]. Comprehensive and effective nursing intervention before and after surgery can effectively reduce the postoperative complications and help patients recover quickly [5]. With the development of endoscopes and auxiliary equipment, colonoscopy has made great progress in the diagnosis and treatment of colorectal diseases [6]. Colonoscopy can not only make correct judgments on various colorectal diseases but also becomes more and more important in terms of treatment [7]. In the past, the diagnosis of colorectal diseases mainly relied on barium enema, but the accuracy was not high, smaller lesions were difficult to find, and sometimes larger lesions were difficult to diagnose [8]. Colonoscopy can not only correctly judge various colorectal diseases but also becomes more and more important in the treatment [9].

With the development of computer technology in recent years, computer-assisted colonoscopy diagnosis technology is also constantly developing. It can provide doctors with powerful clinical help and has a very important application in guiding colonoscopy in the analysis and judgment of lesions [10]. Some colon polyps are proliferative changes, and some are adenomas [11]. Some polyps, such as papillary polyps and colon polyps, have a high carcinogenesis rate, and colorectal cancer is one of the deadliest but preventable malignancies [12]. In recent years, it has become one of the deadliest diseases in the world [13]. The mortality rate of colorectal cancer is only lower than that of lung cancer [14], and it has been recognized that adenomatous polyps may be cancerous. According to statistics, carcinogenesis occurs in large villous adenomas [15]. If colorectal cancer can be detected at an early stage, it is a change in the cure rate [16]. Colitis is also a common colon disease, and different degrees of colon erosion and bleeding can be seen under a colonoscope [17]. Colitis is divided into nonspecific inflammation and specific inflammation. The clinical manifestations are abdominal pain, diarrhea, or blood in the stool, which brings great pain to the patient. How to use computers to analyze colonoscopy images is the ultimate goal of our research [18]. Image segmentation plays an increasingly important role in medical image processing and analysis, and it has a wide range of applications in a large number of medical research and applications such as tissue volume calculation, diagnosis, disease location, anatomical structure research, and computer-assisted surgery [19]. Although modern imaging methods provide more accurate tissue structure segmentation, accurate segmentation of ultrasound image is still a big challenge. This is because ultrasound image is often interfered by noise and sampling errors. If the edge detection or threshold method is not effective, postprocessing is usually required to remove meaningless object boundaries [20]. The method used in the study can obtain better segmentation results for colon polyp images.

Under the ultrasonic imaging and endoscopic resection of intelligent segmentation algorithm, whether nursing intervention can promote the good recovery of patients with colon polyps was explored in this study. Patients with colon polyps were selected and divided into an experimental group and a control group. The colonoscopy polyp ultrasound images were preprocessed to select the seed points and background points, and the random walk decomposition algorithm was adopted to calculate the probability of each marked point and output the marked image. This study can reduce the adverse reactions of patients after surgery, lower the possibility of postoperative mucosal perforation and postoperative complications, allow the patient to recover quickly, and further improve the patient's life comfort.

## 2. Materials and Methods

### 2.1. Research Objects

A total of 180 patients were included in this study from February 2018 to December 2020, including 90 in the experimental group and 90 in the control group. Among the patients, 93 were males and 87 were females, and the average age was 53.26 ± 3.74 years old.

The inclusion criteria were defined as follows: patients who met the conditions for diagnosis of this disease, patients who were 19~ 65 years old, and patients who had signed the written informed consents. The exclusion criteria were defined as follows: patients with inability to speak, audiovisual disability, and mental illness; pregnant and lactating patients; patients with hyperthyroidism, hypothyroidism, immune problems, blood diseases, trauma, fractures, and other diseases that affected exercise and caused damaged visceral motor nerves; patients with severe heart, lung, liver, and kidney diseases, combined with severe organ diseases such as the heart, liver, and kidney, malignant tumor diseases, and immune diseases before the surgery; and patients with abdominal effusion. The discontinuation criteria were described as follows: serious adverse events and feelings were found during the treatment; and the loss rate of subjects during the experiment was >19%.

In this study, a total of 180 patients met the above inclusion and exclusion criteria. This study had been approved by the Medical Ethics Committee of Hospital, and the family members of the patients included in the study had signed the consent forms.

### 2.2. Ultrasound Scan

The Color Doppler ultrasound diagnostic apparatus was adopted, which was equipped with I31-6 linear array probe (6 ~ 13 MHz). The scanning gap was determined by using the spontaneous aiming method. A monitoring point was set at the level of the abdominal aorta on the top of the diaphragm before starting the monitoring scan. When the observation point threshold became 149 hu, the scan started, and the scan delay time was 7.3 s. The scan area was from above the diaphragm to the level of the iliac crest. The venous phase scan was performed 29 s after the beginning of the arterial phase, and the patient held his breath during the scan (the patient was trained to hold his breath before the scan). The double-barrel automatic high-pressure syringe was adopted to inject 79-91 mL through the anterior elbow joint. The injection flow rate was 4.9 mL/s, and the injection was flushed with 18 mL of normal saline. The scanning parameters were defined as follows: tube voltage was 119 kV, the tube current was 287 mAs, the collimation was 135 layers × 0.735 mm, the rotation time was 0.45 s/r, the spacing was 0.887, matrix was 543 × 543, and the reconstruction algorithm was standard (A).

A nonemergency patient was required to fast for 3 ~ 7 hours. The noncooperative nonemergency patients had to be sedated and hypnotized. Emergency patients did not make special preparations. After the routine abdominal scan in the supine position, the ascending colon, transverse colon, descending colon, sigmoid colon, and rectum were scanned with linear array probes. When a suspicious lesion was found, the lesion had to be enlarged to carefully observe the shape, size, internal echo, and blood supply of the lesion, and measure the size. All patients were followed up for colonoscopy, postoperative diagnosis, and pathological examination after ultrasound.

### 2.3. Image Decomposition Using Intelligent Algorithm

The flow chart of colonoscopy polyp image processing is shown in Figure 1. Seed points and background points were selected for preprocessing. For images, the random walk was adopted to calculate the probability from each point to each mark point, then determine which mark point each point belongs to, and finally output the marked image. Figure 1 showed the image processing process of colonoscopy polyp lumps.

The seed points and background points cannot be too small; otherwise, it will cause inaccurate segmentation. If too many seed points and background points were selected, the results would hardly improve, and it was easy to produce incorrect segmentation results and inaccurate results. Therefore, the conditions of seed points and background points were selected in this study.

In addition, the image segmentation algorithm of fuzzy connectivity combined with similarity test was applied in this study to detect the polyps. The tumor images were processed, the fuzzy correlation degree and maximum value of each point and seed points were calculated, and the optimal path was determined. Then, the attribute similarity between each point on the path and the seed points was defined to get the optimal path. The diameter was calculated. The attribute similarity of the seed points should be greater than the threshold to ensure that the attributes of the points in the area were similar to the attributes of the seed points. However, the calculation time of this algorithm was too long, it had to determine a threshold value after the similarity between each point, and the seed points were calculated. However, the similarity difference among most images was very small, which made it difficult to obtain a suitable segmentation result. If *x* samples *n*_*i*_ ∈ *D*^*X*^ (*i* = 1, 2 ⋯ *x*) was controlled into *q* types, then the equation below could be obtained:

(1) $$\begin{array}{c} U_{\text{Il}}=\left\{1^{1\text{st}}2^{\text{Other}}\right.. \end{array}$$

The properties of matrix *U* can be expressed as *U* = (*U*_*il*_).

(2) $$\begin{array}{c} U_{il}\in \left(1,2\right),\\ \overset{e}{\underset{i=1}{\sum }}U_{il}=2\left(l=2,3,\cdots x\right). \end{array}$$

The overall difference was expressed as

(3) $$\begin{array}{c} P\left(U\right)=\overset{e}{\underset{i=1}{\sum }}P^{\left(l\right)}\left(u\right)=\overset{e}{\underset{i=1}{\sum }}\overset{e}{\underset{l=1}{\sum }}U_{il}\left\|n_{l}-‾n_{i}\right\|. \end{array}$$

In the above equation, *w* was the vector of current components, *l* is the current source, *d* was the voltage source, and *q* represented the voltage potential. These can be combined into a linear system:

(4) $$\begin{array}{c} B^{F}DAs+B^{F}Zq=\text{l}. \end{array}$$

How to determine the closing value is very important, but now it is difficult to get a good segmentation effect by automatically selecting the threshold. Manually selecting the closing value to obtain the segmentation result showed that the segmentation effect was relatively poor. Therefore, this method was inconvenient for the segmentation of colonoscopy images with a lot of noise.  Figure 2 showed the similarity between each point and seed points.

The whole point set randomly walked on *f* = {0, 1, ⋯*n*}, where 0 and *n* points were absorption walls; that is, when the particle reached 0 or *n*, it only stayed at this point and stopped random wandering process. *D*(*y*) showed the starting point and then reached to the point *n*. Therefore, the properties of *D*(*y*) were as follows:

(5) $$\begin{array}{c} D\left(0\right)=0,\\ D\left(n\right)=2,\\ D\left(y\right)=\left(\frac{2}{3}\right)D\left(y-2\right)+\left(\frac{2}{3}\right)D\left(y+2\right). \end{array}$$

It was considered that the point set definition was called reconciliation when it was satisfied. Therefore, the moving randomly on a straight line was essentially to find the sum of the two endpoints and the setting of the harmonic function theorem was defined to take the maximum and minimum values at the dividing point. The theorem that sum was a harmonic function defined on a set of points was commonly used in this equation.

### 2.4. Surgery Methods

Firstly, a gauze pad (slightly larger than the electrode plate) was moistened with normal saline, placed on the electrode plate, attached on the patient's calf or gastrocnemius muscle, and then fixed with a lace. Secondly, the high-frequency power switch was turned on, and different current intensities (index or *W*) were selected according to the size of the polyp, especially the size of the polyp pedicle. The assistant held the handle of the electric snare and handed the end of the electric snare to the operator. The operator inserted the electric snare into the hole of the endoscopic biopsy forceps and sent the electric snare to the vicinity of the polyp. The assistant can push out the electric snare, and the operator can clamp the polyp pedicle 3-4 mm away from the mucosal surface, so that the assistant can tighten the snare and strangle the polyp pedicle. However, excessive force should be avoided to cause bleeding after polypectomy. The operator intermittently stepped on the electrocoagulation foot brake pedal for a few seconds. When the base turned white, the power switch was depressed for a few seconds and the ferrule was tightened to cut off the polyp. During the operation, the endoscope and the high-frequency generator should be reliably connected to the ground wire to ensure the safety of the patient and the surgeon. The cut polyp was targeted, the electric attraction switch was stepped on, and the endoscope attraction button was pressed to make the polyp adsorb to the end of the endoscope. After the operation, the wound should be carefully observed for bleeding. If necessary, adrenaline at 1 : 10000 was sprayed locally through the endoscope or stop bleeding with a coagulation electrode.

### 2.5. Perioperative Nursing Method

Preoperative nursing method was described as follows. Patients in the control group were given conventional nursing, and those in the experimental group were given surgical treatment. The comprehensive nursing methods before, during, and after the surgery were described as follows. It was recommended that the patient eat one meal 3 days before the surgery and reduce the amount of semiliquid food 1 night before the operation and 7 hours before the operation. It had to provide effective psychological counseling to the patient before the surgery and introduce in detail the operation method, process and method necessity, and relevant precautions. Patients in the recovery period of similar operations can be invited to the site to explain, so as to reduce the anxiety and psychological pressure of the patients due to the surgery and improve the degree of cooperation during the surgery. Nurses before surgery should actively communicate with patients, give meticulous nursing, and ask about their medical history, physical condition, and other basic information. The colonoscopy was explained to the patient in detail; the operation steps, links, and possible problems of the resection were explained to the patients to reduce the occurrence of complications and improve the patient's compliance with the surgical treatment. The patients were assisted to hold hands, determine the surgical position, and perform the venous access, electrocardiograph (ECG) monitoring, and oxygen inhalation.

During the surgery, the patient had to actively cooperate with the doctor, assist the doctor to insert the lens, and adjust the position correctly to make the field of vision clearer. It had to pay attention to gentle movements to prevent intestinal wall damage. The occurrence, discovery, and arrival of polyps should follow the doctor's instructions and do a good job of trap management. If the snare was too tight, the polyp pedicle was very thin, and when it was not charged, because there was no electrocoagulation, mechanical severance, and bleeding were prone to occur. After polyp resection, the patient had to stand up to find the difficulty of intestinal cavity. It should check and confirm that the residual pedicle was normal. The specimen was fixed in 10% formaldehyde solution and compared with the pathological results. Finally, the specimen was sent to the pathology department for inspection.

Patients are prone to acute bleeding within 1 hour after surgery. If it is caused by mechanical cutting or electric cutting current, norepinephrine can be sprayed for management. Delayed bleeding is prone to occur 1 hour after surgery, mainly due to too long electrocoagulation time; if it is caused by too long or excessive postoperative activity time, dietary intervention and nursing work and rest guidance should be given. The rest time should be determined according to the patient's condition; 6 hours on bed and no physical work within 1 week had to be ensured. It should avoid severe coughing and bowel movements to avoid increased abdominal pressure. Patients with polyps > 1.0 cm or bleeding at risk of perforation should stay in bed for about a week and no major surgery within one month. The patient was not allowed to eat for 6 hours after the surgery. After 24 hours, the patient can eat more liquid and semiliquid food according to the improvement of the condition and gradually transit to a normal diet, and no irritating food was allowed within one week. Perforation is the most serious postoperative complication. Blood pressure, heart rate, and other vital signs should be monitored comprehensively. Adverse reactions such as abdominal pain and blood in the stool should be treated promptly as directed by the doctor.

### 2.6. Observation Indicators

The occurrence of complications between the two groups of patients should be observed and compared carefully. It had to observe the physiological indicators of the patients, track the patients' discomfort symptoms, and take emergency measures. The main indicators included mucosal perforation, blood in the stool, abdominal pain, and small bleeding situation.

### 2.7. Statistical Analysis

The SPSS18 software was adopted to complete statistics. Counting data were expressed as a rate (%). The mean of two pairs of continuous variable data was compared by *t*-test, and the mean of continuous variable data was analyzed by variance analysis and chi-square test. *P* < 0.05 indicated that the difference was statistically significant.

## 3. Results

### 3.1. Basic Data of Patients

A total of 200 cases were collected in this study, and 20 cases were excluded according to the exclusion criteria. Finally, a total of 180 patients were included in this study, including 90 in the experimental group and 90 in the control group. A total of 132 patients undergoing colon polyp resection in our hospital from June 2017 to June 2018 were selected as the research subjects. All patients were clinically diagnosed with colon polyps and treated with colonoscopic electrocoagulation and resection. There were 93 males and 87 females with the average age 53.26 ± 3.74 years old. They were randomly divided into an experimental group and a control group.  Table 1 showed the basic data of patients.

### 3.2. Evaluation of Ultrasound Image Segmentation Effect Based on Intelligent Segmentation Algorithm

Colon polyp segmentation is a part of the digital simulation colon surgery planning system and is a system that can assist in the treatment of colon diseases. In this study, the quantitative analysis of the segmentation results of colonoscopy polyps and tumors mainly used experimental methods to analyze the performance of the algorithm; that is, the performance of the segmentation algorithm used was determined by studying the results of image segmentation. The accuracy of intelligent segmentation algorithm reached 81%.  Figure 3 below showed the ultrasound image of intestinal polyps and the result of segmentation of the target region in the ultrasound image by the algorithm.

### 3.3. Comparison on Nursing Effect Evaluation Indicators

The incidence of complications in the experimental group was 4.83%, which was lower than 16.66% in the control group, and the difference was statistically remarkable (*P* < 0.05). The comparison on the mucosal perforation for patients in the control group and the experimental group after surgery is shown in Figure 4. The number of patients with mucosal perforation in the experimental group was 1, while that in the control group was 2, and the difference was statistically obvious (*P* < 0.05).

The postoperative blood in the stool comparison of patients in the two groups was compared, and the results are illustrated in Figure 5. The number of blood in the stool in the experimental group was 2 and that in the control group was 4. The difference was statistically visible (*P* < 0.05).

The postoperative abdominal pain of patients in two groups was compared, and the results are given in Figure 6 below. The numbers of patients with abdominal pain in the experimental group and the control group were 2 and 7, respectively, showing obviously statistical difference (*P* < 0.05).

The postoperative small bleeding of patients in two groups was compared, and the results are given in Figure 7 below. The numbers of patients with small bleeding in the experimental group and the control group were 1 and 2, respectively, showing obviously statistical difference (*P* < 0.05).

## 4. Discussion

High-frequency electrocoagulation has been widely used in the treatment of colon polyps due to its short operation time, accurate positioning, and easy operation [21]. Comprehensive nursing intervention can effectively improve the success rate of colon polyp resection under colonoscopy [22]. Nursing measures such as the quality of the patient's preoperative bowel preparation directly affect the clinical diagnosis and treatment and the occurrence of complications. Those patients whose intestinal cleanliness is lower than Grade B need to be prepared and scheduled for surgery again. Insufficient bowel preparation can easily lead to missed diagnosis and misdiagnosed, as well as complications such as bleeding and perforation. In addition, the unclean intestinal cavity seriously affects the operator's mood and patience and has a certain interference effect on the operation. During the surgery, the cooperation of nurses is very important. Some polyps are located behind the colon folds and can only be revealed by changing the patient's position or rotating the mirror body [23]. The ultimate goal of this study was that the entire system of the colonoscopy image analysis system should include preprocessing, image segmentation, and feature classification.

Image segmentation is a difficult point in image processing [24]. Many people have made different progress in this regard. When various methods are applied in actual projects, different problems will always be encountered. Colonoscopy images are known for their variability and complexity of noise. Using automatic segmentation to achieve fine segmentation is a difficult point. Colonoscopy computer-aided diagnosis system shows high requirements for image segmentation, and the method currently used is manual intervention, whether it is random walk or single-mean clustering [25]. In the process of processing the polyp mass image, the seed points and background points in the image are manually selected. The erosion and bleeding images are also preset to achieve segmentation. It has to explore further on how to improve the realization of automatic segmentation. The weight of the random walk method is the component in each color space [26]. Although the segmentation effect is ideal, if other image texture information is used, the segmentation effect will be better for different images and lesions. In this study, intelligent algorithms were adopted to process ultrasound images of colon polyp patients, and the results showed that the accuracy of intelligent segmentation algorithm reached 81%. The incidence of complications in the experimental group was 4.83%, which was lower than 16.66% in the control group (*P* < 0.05). It showed that the application of artificial intelligence technology in the field of medical image processing can achieve excellent results, which was similar to the results of Dumoulin and Hildenbrand [27]. The segmentation work in this study was only an important part of the entire analysis system, but the process of feature classification analysis and judgment had to continue to complete the colonoscopy automatic analysis system, and there is still a lot of work to be done. Therefore, patients have to be regularly reviewed and strictly followed up [28]. Under the ultrasonic imaging and endoscopic resection of the intelligent segmentation algorithm, nursing intervention treatment promotes the good recovery of patients with colon polyps.

## 5. Conclusion

In order to explore the effect of artificial intelligence technology in the ultrasound image processing of colon polyp disease and to provide a basis for improving clinical diagnosis and treatment, the artificial intelligence algorithms were adopted to realize the recognition of the region of interest in the image. In summary, fine nursing throughout the entire process of endoscopic polypectomy can effectively reduce the complications of colon polyp resection and improve the quality of clinical nursing. Perioperative refined nursing intervention for colon polyp patients undergoing endoscopic electrosurgical resection can decrease postoperative adverse reactions; reduce postoperative mucosal perforation, blood in the stool, abdominal pain, and small bleeding; lower the incidence of postoperative complications; and allow patients to recover quickly, enhancing the life comfort of patient. There were also many shortcomings in the study. Firstly, it was found in practice that the image quality of colon polyps was getting better and better, but it failed to measure the specific data of all patients in this study due to incomplete data. Therefore, the difference between the experimental group and the control group cannot be fully analyzed. In this study, the sample size was too small and should include more experimenters.

## Figures and Tables

**Figure 1:** Image solution for colonoscopy polyps.

**Figure 2:** Image sample of the similarity between each point and seed points.

**Figure 3:** The ultrasound image of colon polyps and the result of the algorithm segmentation of the target region in the ultrasound image.

**Figure 4:** Comparison on the number of mucosal perforation patients in the two groups.

**Figure 5:** Comparison on the number of patients with blood in the stool in the two groups.

**Figure 6:** Comparison on the number of patients with abdominal pain in the two groups.

**Figure 7:** Comparison on the number of patients with small bleeding in the two groups.

**Table 1:** Basic data of patients.

	Experimental group (%)	Control group	*P* value
Age (years old)	55 ± 2.4	50 ± 12	*P* > 0.05
Gender			
Males	58.4%	58.3%	*P* > 0.05
Females	41.6%	41.7%	

## Data Availability

The data used to support the findings of this study are available from the corresponding author upon request.
